# Hemorrhagic Infarct as a Rare Presentation of Vascular Ehlers-Danlos Syndrome in a 40-Year-Old Female: A Case Report

**DOI:** 10.7759/cureus.76952

**Published:** 2025-01-05

**Authors:** Wahab Moustafa, Taranpreet Singh, Arzoo Siddiqi, Anoushka A Sehgal, Bismil Afghan

**Affiliations:** 1 Neurosurgery, SRH Wald-Klinikum Gera, Gera, DEU; 2 Internal Medicine, Mahatma Gandhi Mission (MGM) Medical College and Hospital, Navi Mumbai, IND; 3 Internal Medicine, Dow University of Health Sciences, Karachi, PAK; 4 Internal Medicine, Mahatma Gandhi Medical College and Research Institute, Pondicherry, IND; 5 Internal Medicine, Nishtar Medical University, Multan, PAK

**Keywords:** col3a1 mutation, connective tissue disorder, genetic testing, hemorrhagic infarct, vascular ehlers-danlos syndrome

## Abstract

This case report presents a 40-year-old female with vascular Ehlers-Danlos Syndrome (vEDS) who presented with acute right-sided weakness and altered consciousness due to a rare hemorrhagic infarct in the left middle cerebral artery (MCA) territory. Initial examination revealed severe neurological impairment and subtle signs of connective tissue disorder, including skin hyperextensibility and joint hypermobility. Imaging confirmed a hemorrhagic infarct, while laboratory findings showed leukocytosis, anemia, and hypokalemia. Given her family history and clinical features, genetic testing confirmed a *COL3A1 *mutation diagnostic of vEDS. Management included blood pressure control, potassium replacement, and intracranial pressure reduction, followed by a long-term care plan. This case emphasizes the importance of considering vEDS in atypical vascular presentations and highlights the value of genetic testing in diagnosing this high-risk condition.

## Introduction

Ehlers-Danlos Syndrome (EDS) represents a group of inherited connective tissue disorders collectively affecting approximately 1 in 5,000 individuals worldwide [1]. Of the 13 identified subtypes, hypermobile, classical, and vEDS are among the most common. Characterized by joint hypermobility, skin hyperextensibility, and tissue fragility, EDS manifests with a range of symptoms that vary significantly among patients [2]. The condition affects individuals across all ethnic groups and genders, with certain subtypes showing higher prevalence in females. Typically, symptoms emerge in childhood, though they may develop at any age, often complicating early diagnosis. The clinical presentation, family history, and genetic testing, based on the 2017 International Classification of EDS criteria, collectively aid in establishing a definitive diagnosis [3].

Vascular Ehlers-Danlos Syndrome (vEDS), though rare, is recognized as the most severe form of EDS, affecting an estimated 1 in 50,000 to 1 in 200,000 individuals [2]. This subtype is characterized by thin, translucent skin, pronounced arterial and organ fragility, and characteristic facial features, often identifiable upon examination. A hallmark of vEDS is vascular fragility, which clinically manifests as spontaneous arterial rupture, often occurring without prior trauma and involving critical structures such as the lungs, gastrointestinal tract, or brain. Such events carry a high mortality risk due to the sudden and unpredictable nature of complications. Genetic testing confirming mutations in the COL3A1 gene is essential for diagnosing vEDS, as it establishes the underlying cause of these life-threatening manifestations. Cerebrovascular complications, including cerebrovascular accident (CVA) with hemorrhage leading to hemorrhagic infarct, are among the rarest yet deadliest outcomes in vEDS [3]. Management is primarily preventative, emphasizing the minimization of physical trauma, meticulous blood pressure control, regular cardiovascular imaging, and genetic counseling [4]. Emergency planning for potential vascular events further highlights the critical need for vigilant care, as vEDS remains the most dangerous form of EDS due to its elevated risk of sudden, life-threatening complications.

This case report aims to underscore the clinical complexity and diagnostic challenges associated with vEDS, particularly in cases presenting with rare complications such as hemorrhagic infarcts. By examining the clinical journey of a 40-year-old female with vEDS, this report highlights the need for a high index of suspicion for connective tissue disorders in atypical vascular presentations. Through detailed clinical, genetic, and imaging insights, the objective is to illustrate the critical importance of early diagnosis, vigilant monitoring, and tailored management strategies in preventing fatal outcomes in vEDS patients. Additionally, this case serves as a valuable reference for clinicians in recognizing the subtle yet high-risk manifestations of vEDS, reinforcing the essential role of genetic testing in confirming the diagnosis and guiding comprehensive, multidisciplinary care.

## Case presentation

A 40-year-old female presented to the hospital with a primary complaint of sudden onset right-sided body weakness and an altered level of consciousness lasting approximately four hours. Her medical history revealed a long-standing diagnosis of hypertension (10-15 years), managed with antihypertensive medication but with noted poor compliance, which may have contributed to sporadic blood pressure control. The patient reported being in her usual state of health prior to the incident but developed an abrupt, progressive weakness on the right side of her body, affecting both the upper and lower limbs simultaneously. This weakness quickly progressed to a complete loss of motor power on the affected side. Within an hour, her neurological status deteriorated further, with initial symptoms of confused speech that escalated to a total loss of consciousness.

Upon arrival at the hospital, a neurological examination showed a Glasgow Coma Scale (GCS) score of E2V1M4, totaling 7/15, indicating a severely impaired level of consciousness. Central nervous system examination revealed bilateral upgoing plantar reflexes, mid-dilated pupils reactive to light, and brisk reflexes in the right upper and lower limbs, suggesting significant neurological compromise. Additional examination of her skin and joints uncovered findings indicative of a connective tissue disorder: her skin exhibited marked hyperflexibility, her joints demonstrated pronounced hypermobility, and there was evidence of hyperfragility, as indicated by a dislocation of the right knee joint. A Beighton score evaluation was performed to further assess joint hypermobility, yielding a score of 2/9. While this low score did not strongly suggest generalized joint hypermobility, it did not rule out vEDS, given the patient’s clinical presentation and family history. The patient disclosed that she was married to her cousin, and further family history revealed a background of other congenital disorders, increasing the suspicion of an underlying genetic disorder.

A structured diagnostic approach was implemented, beginning with baseline laboratory tests and a non-contrast computerized tomography (CT) scan of the brain to differentiate between potential hemorrhagic and ischemic causes of her acute neurological presentation. Significant findings in her baseline results included elevated white blood cell (WBC) count (17.5 x10^9^/L), indicative of a possible underlying infective process, a low hemoglobin level (10.66 g/dL), and marked hypokalemia (2.41 mmol/L), which required immediate correction. Urinalysis revealed notable proteinuria (3+) and an elevated red blood cell count (10-15/hpf), suggesting additional renal involvement or systemic implications of her condition. These abnormalities informed the initial management steps, including antibiotic administration and potassium replacement therapy, alongside imaging to clarify the cause of her neurological deficits. A summary of significant baseline findings is provided in Table 1.

**Table 1:** A summary of the significant baseline findings. WBC: White blood cell; g/dL: Grams per deciliter; mmol/L: Millimoles per liter; RBCs: Red blood cells; hpf: High-power field

Investigation	Result	Reference Range
WBC Count	17.5 x10^9^/L	4-11 x10^9^/L
Hemoglobin	10.66 g/dL	13-18 g/dL
Potassium	2.41 mmol/L	3.5-5 mmol/L
Protein (Urine)	3+	<150 mg/d
RBCs (Urine)	10-15 /hpf	<3 RBCs/hpf

CT brain imaging revealed a large hypodense area within the left frontal and parietal lobes, consistent with an acute to subacute infarct in the territory of the left middle cerebral artery (MCA), measuring approximately 6-7 cm (Figure 1). A mild mass effect was noted, causing sulcal effacement and slight compression of the left lateral ventricle, accompanied by a midline shift. A surrounding hyperdense area was also observed, suggesting hemorrhage into the infarcted region.

**Figure 1:** The CT brain showing mass effect with compression of left lateral ventricle, with accompanied midline shift. The lesion is being represented by the arrow.

The patient’s management plan initially focused on stabilizing her acute condition. Mannitol was administered to reduce intracranial pressure, and systolic blood pressure was carefully maintained between 160-180 mmHg over the next 72 hours. Antihypertensive therapy was adjusted to manage her chronic hypertension more effectively, and potassium supplementation was initiated to correct the documented hypokalemia. Concurrently, antibiotics were given to address the suspected underlying infection.

Given her unique clinical presentation, with notable hypermobility, hyperflexibility, and joint dislocations, further inquiry with her family revealed a long-standing history of joint instability and skin changes. This led to a high suspicion of EDS, particularly vEDS, due to her severe vascular complications. A Beighton score assessment for hypermobility was performed, yielding a score of 2/9, which, while low, did not rule out vEDS given the specific clinical picture. Genetic testing was subsequently conducted, confirming a mutation in the COL3A1 gene, thus establishing the diagnosis of vEDS.

As vEDS has no curative treatment and management is primarily supportive, the patient was given a comprehensive care plan aimed at reducing the risk of future vascular events. This included a tailored physical therapy regimen to strengthen her right-sided motor function and improve her overall mobility while minimizing strain on fragile tissues. She was also educated on preventive measures, such as avoiding high-risk activities, maintaining blood pressure control, and engaging in regular cardiovascular monitoring. Genetic counseling was recommended for her family, considering the hereditary nature of vEDS.

At present, the patient’s neurological status shows gradual improvement, with a slowly increasing GCS score. Physical therapy is ongoing to aid in the recovery of motor function in her right upper and lower limbs. Given the high risk of recurrent vascular complications associated with vEDS, regular follow-up is planned to monitor her condition closely.

## Discussion

This case report describes a rare and complex manifestation of vEDS in a 40-year-old female, illustrating the severe complications that can arise in this condition. Vascular EDS is the rarest and most severe form of EDS, affecting approximately 1 in 50,000 to 1 in 200,000 individuals, with a median survival age of 48 years [4]. Although our patient’s age aligns with the typical presentation of vEDS, which can manifest at various life stages, her development of a hemorrhagic infarct stands out as an uncommon and life-threatening presentation. Vascular complications, including spontaneous arterial and organ rupture, are hallmarks of vEDS, but cerebrovascular events such as hemorrhagic infarcts remain among the rarest and most severe of these manifestations [5]. This case thus emphasizes the need for clinicians to recognize the neurovascular risks associated with vEDS, even when initial assessments may not immediately point toward a connective tissue disorder.

The clinical presentation in our patient, marked by hyperextensible skin, joint hypermobility, and tissue fragility as evidenced by a knee dislocation, aligns with the diagnostic characteristics of vEDS. However, these features can vary significantly among individuals with vEDS. Notably, genetic testing confirmed a mutation in the COL3A1 gene, which is fundamental for diagnosing vEDS and is considered a standard criterion [6]. Genetic confirmation is particularly vital for vEDS, given its potentially fatal vascular complications, and can help guide both acute management and preventive care strategies for affected patients and their families.

A distinctive feature in this case is the patient’s low Beighton score of 2/9, which indicates mild joint hypermobility. Although joint hypermobility is common in many subtypes of EDS, it is generally less pronounced in vEDS, often leading to diagnostic challenges when evaluating patients solely based on hypermobility scores. This highlights the importance of not excluding vEDS based solely on a low Beighton score, as other clinical indicators, such as tissue fragility and vascular symptoms, may still point toward this diagnosis [6]. This case underscores the value of a thorough clinical evaluation in suspected vEDS patients, including skin and joint assessments, family history, and, when warranted, genetic testing to confirm diagnosis despite subtle features.

The pedigree chart demonstrates the family history of the patient diagnosed with vEDS. It highlights the consanguineous marriage between the patient and her first cousin, reflecting a shared genetic lineage through their common grandparents. This familial relationship significantly increases the likelihood of inheriting recessive genetic mutations, which may have contributed to the patient’s presentation. The chart also includes the offspring of the couple, emphasizing the importance of genetic counseling to evaluate the risk of vEDS and other hereditary disorders in their children. This visual representation in Figure 2 underscores the relevance of family history and consanguinity in understanding the genetic predisposition to vEDS.

**Figure 2:** Pedigree chart illustrating consanguinity and genetic context in a patient with vascular Ehlers-Danlos syndrome.

Management of this patient balanced acute intervention with a long-term care approach. Addressing the acute complication of hemorrhagic infarction involved immediate stabilization, while preventive strategies targeted the reduction of recurrent vascular risks. This dual approach is essential in managing vEDS, given the disorder’s propensity for sudden and life-threatening vascular events [7]. Furthermore, integrating physiotherapy into the management plan highlights the importance of addressing musculoskeletal health in vEDS patients. Physiotherapy aims to improve function without overstraining the fragile tissues inherent to vEDS, and it can help maintain joint stability and mobility, thereby enhancing quality of life.

To establish the diagnosis of vEDS, genetic testing was performed using DNA extracted from the patient’s peripheral blood. The analysis, outsourced to a certified genetic laboratory, involved whole-exome sequencing (WES) followed by targeted Sanger sequencing to confirm the results. This identified a heterozygous pathogenic mutation in the COL3A1 gene, a hallmark of vEDS. The mutation was classified as pathogenic based on the American College of Medical Genetics and Genomics (ACMG) criteria, which included its prior documentation in the OMIM database and functional evidence from the literature. Segregation analysis using DNA from the patient’s immediate family revealed an autosomal dominant inheritance pattern, aligning with the typical genetic mechanism of COL3A1 mutations. These findings confirmed the diagnosis and underscored the genetic etiology of her condition.

It is noteworthy that the genetic testing, while critical for this patient, was not covered by the national healthcare system and had to be paid for by the patient. This highlights the financial burden associated with diagnosing rare disorders, particularly in resource-limited settings, and underscores the need for broader access to genetic testing in such populations.

This case underscores the critical importance of early recognition and diagnosis of vEDS, especially in patients presenting with atypical vascular complications. Genetic testing played a key role in confirming the diagnosis, while the tailored management plan incorporated both acute care and preventive strategies and served as a model for managing vEDS patients effectively. Future research into targeted treatments for vEDS is necessary to improve outcomes and reduce the risk of severe complications in this high-risk population.

## Conclusions

This case report highlights the critical need to consider vEDS in patients presenting with severe vascular events, particularly when initial symptoms may not obviously indicate a connective tissue disorder. The rare occurrence of a hemorrhagic infarct in this 40-year-old female with vEDS emphasizes the high potential for life-threatening neurovascular complications in this population. Comprehensive clinical assessment, including evaluation of skin and joint abnormalities even in acute settings, proved essential in identifying subtle signs of vEDS. Genetic testing played a pivotal role in confirming the diagnosis, underlining its value when clinical features are atypical. In this case, the management approach balances immediate intervention with long-term preventive strategies and serves as a valuable model for handling complex vEDS cases. This report underscores the importance of maintaining a high index of suspicion for vEDS in patients with unexplained vascular events and highlights how early recognition and targeted care can substantially improve patient outcomes. Future research on effective treatments and preventive measures for vEDS remains crucial in reducing the burden of this challenging condition.
